The article "Nanohydroxyapatite Hydrogel Can Promote the Proliferation and Migration of Chondrocytes and Better Repair Talar Articular Cartilage" was published in 2022. Journal: Comput Math Methods Med.

# Nanohydroxyapatite Hydrogel Can Promote the Proliferation and Migration of Chondrocytes and Better Repair Talar Articular Cartilage

**DOI:** 10.1155/2022/8388473

**Published:** 2022-05-26

**Authors:** Yuxuan Zhang, Yi Cui, Jian Tian, Xueming Chen, Tonglong Xu, Jiajia Liu, Yajun Xu

**Affiliations:** ^1^Department of Foot and Ankle Surgery, Wuxi No.9 People's Hospital Affiliated to Soochow University, Wuxi, 214000 Jiangsu Province, China; ^2^Department of Orthopedics, Yancheng First People's Hospital, Affiliated Hospital of Nanjing University Medical School, Yancheng, 224000 Jiangsu Province, China; ^3^Department of Emergency, Affiliated Hospital of Nantong University, Nantong, 226000 Jiangsu Province, China

## Abstract

As an important load-bearing part of the body, joints are prone to articular cartilage degradation during exercise, resulting in joint pain, swelling, and deformity, which has an adverse impact on patients' life quality and social medical security. Therefore, this study aims to test an effective biopolymer scaffold in promoting the growth of chondrocytes in talus. Hydrogel (Gel)-nanohydroxyapatite (nHA) was invented as a new type of biopolymer scaffold for osteoarthritis treatment in this research. To detect the effects of Gel-nHA on guidance, cartilage matrix secretion, mineralization, proliferation, and migration of chondrocyte, we cultured chondrocytes to study the biological properties of nHA. It was found that Gel could guide chondrocytes to permeate and migrate, so it could be used as acellular matrix scaffolds for chondrocyte regeneration. In addition, nHA could stimulate chondrocytes to secrete cartilage matrix, such as type II collagen and mucopolysaccharide (GAGs). At the same time, nHA help to induce chondrocyte mineralization and stimulate the secretion of type X collagen, so as to better maintain the integrity of bone cartilage interface. In Gel-nHA, chondrocyte viability could be better maintained, and the proliferation and migration of chondrocytes could be better promoted, so as to better repair the articular cartilage of talus. Therefore, the Gel-nHA scaffold is expected to become an effective method for repairing talus cartilage in the future.

## 1. Introduction

In the human movement system, joints can integrate bones and bones completely and complete various movements such as flexion, extension, and rotation with the help of muscles, so as to maintain the stability and flexibility of the body [1]. Articular cartilage, as the cartilage tissue covering the joint surface, is of great significance in reducing the load-bearing pressure, increasing the stress area, and lubricating the joint [2], so as to effectively protect the articular surface and maintain the normal movement of the joint. As the most frequently used joint in daily life and work, ankle joint should not only bear the heavy pressure of the body, but also bear the daily walking and movement [3]. As a result, articular cartilage of talus is easily damaged due to trauma, joint degradation, arthritis, and other reasons, resulting in rough joint surface, joint pain, and limited activity, which will seriously affect the life quality of patients. Due to the lack of innervation of blood vessels, lymphatic vessels, and nerves, self-healing ability of articular cartilage is relatively low [4]. Once injured, it often needs surgery for repair treatment. However, surgical treatment is more traumatic and expensive, which will cause a greater economic burden on patients and their families [5]. In recent years, with the development of biological tissue engineering, it provides better choices for the repair of cartilage tissue.

Articular cartilage is responsible for reducing joint friction and effectively loading the pressure during exercise. Articular cartilage can effectively compress and bear weight under heavy pressure, which is closely related to the existence of mucopolysaccharide (GAGs) [6]. GAGs can effectively maintain the elasticity of articular cartilage and improve its ability to bear high compression load [7]. In addition, articular cartilage can withstand high tensile and shear stress during exercise, which is mainly related to the existence of type II collagen [8]. Furthermore, keeping the integrity of bone cartilage interface is an important part in the process of cartilage repair, and it can effectively inhibit the invasion and ectopic mineralization of the bottom bone, so as to maintain the efficient connection between bone and cartilage [9]. The bone cartilage interface is formed by calcified cartilage, which is related to the existence of type X collagen [10]. Therefore, in the process of articular cartilage repair, promoting the regeneration of chondrocytes and the secretion of collagen and GAGs are the necessary conditions. Nanohydroxyapatite (nHA) is the main inorganic component of bone and has excellent bone induction and bone conduction function, which is benefit to the formation of new bone. Otherwise, the smaller particles of nHA can provide a larger specific surface area for the adhesion of chondrocytes, and its good mineralization function can stimulate cartilage cells to secrete calcified matrix, which is conducive to the formation of calcified cartilage at the bone cartilage interface [11, 12]. Furthermore, relevant studies found that it could promote the secretion of chondrocytes matrix (GAGs and collagen) [13]. Therefore, we choose nHA as the biomaterial for cartilage repair. However, in the process of clinical application, it is found that nHA has relatively poor fluidity and high hardness. If it is used alone in the repair of articular cartilage, there will be some problems, such as poor targeting and unable to provide a good growth environment for the proliferation of chondrocytes. Therefore, improving the above problems is of great significance to improve the curative effect of nHA and make it better used in the repair of articular cartilage injury.

Relevant studies have found that when nHA is loaded into the corresponding carrier to form nanocomposites, it can effectively reduce its brittleness and improve the targeted transport, so as to better promote the repair of articular cartilage. In this study, we chose hydrogel (Gel) as an inorganic carrier of nHA. The proliferation and differentiation of chondrocytes are inseparable from the extracellular matrix (ECM) of cartilage. Gel can simulate natural ECM, so that it can be used as a natural medium for chondrocytes [14]. Moreover, it has good biocompatibility, which can effectively maintain chondrocytes viability and promote its proliferation. In addition, the absorbability and fluidity of Gel can effectively encapsulate collagen and various inorganic salts and deliver them to the cartilage defects by injection [15]. Therefore, loading nHA into Gel can effectively overcome the shortcomings of nHA, such as high hardness, relatively fragile, and lack of flexible transmission performance, and smoothly transported to cartilage defect area [16, 17]. In this study, a new biological scaffold was formed by combining Gel and nHA to explore the effect of repairing the articular cartilage.

## 2. Material and Methods

### 2.1. The Preparation of Gel-nHA Scaffold

#### 2.1.1. The Synthesis of N-Carboxyethyl Chitosan (CEC)

1 g chitosan (448869, Sigma-Aldrich, USA) and 1.4 mL 90% acrylic acid (045779, Thermo Fisher Scientific, USA) were dissolved in phosphate buffer (PBS) and heated at 50°C for 72 h, The pH was controlled between 10 and 12 via adding NaOH (1 M). Then this solution was freeze-dried for standby.

#### 2.1.2. The Synthesis of Hyaluronic Acid-Aldehyde (HA-ALD)

2.0 g sodium periodate (C19838, Thermo Fisher Scientific) and 2.0 g sodium hyaluronate (C25177, Thermo Fisher Scientific) were dissolved in 200 mL PBS, and then the mixture was magnetically stirred for 3 h at 26°C away from light. After 10% ethylene glycol (A11591, Thermo Fisher Scientific) was added and magnetically stirred for another 1 h, the above mixture was freeze-dried for standby

#### 2.1.3. The Synthesis of Gel and Gel-nHA Scaffold

The prepared CEC, HA-ALD, and adipic acid dihydrazide (ADH, A0638, Merck, Germany) were mixed in PBS at 26°C under magnetic stir for 1 h to form Gel, then 25% nHA (693863, Merck) by total volume was added in Gel and composed Gel-nHA composite scaffold for standby (Figure 1).

### 2.2. Articular Chondrocytes Culture

In this study, we chose mice articular chondrocytes (CP-M092, Procell, Wuhan, China) for in vitro experiments. The above articular chondrocytes were cultured with complete culture medium of mice articular chondrocytes (CM-M092, Procell) and stored in cell incubator (51032124, Thermo Fisher Scientific, MA, USA), growth conditions: 37°C, 5% CO_2_. The above chondrocytes were cultured in 24-well plates for 24 h.

### 2.3. Adsorption of Gel Scaffold on Chondrocytes

The cultured cells were diluted with phosphate buffer solution (PBS) to 1 × 10^6^/mL, and 500 *μ*L of the above cell solution was inoculated on the Gel surface and then cultured in complete culture medium of human articular chondrocytes for another 24 h. After cleaning with PBS, the cells were fixed with formaldehyde and stained with FITC. Then, the penetration of articular chondrocytes in the Gel was observed by confocal microscope (FV3000, OLYMPUS, Japan), and the scanning layer thickness is 50 *μ*m. Fluorescence spectrophotometer (WHF93, China) was used for fluorescence intensity test.

### 2.4. Cartilage Matrix Detection In Vitro

The Gel and Gel-nHA were added into 6-well plate, respectively. 1-mL cultured articular chondrocyte solution, which was diluted to 1 × 10^4^/mL with PBS, were seeded on the above materials, and then 2-mL complete culture medium of human articular chondrocytes were added in. The above articular chondrocytes act as Gel group and Gel-nHA group. In addition, 1 mL of the above diluted cell solution was added into 6-well plate as control group, and 2-mL similar medium was added in. After being cultured for 14 d, collagen type II, collagen type X, and GAGs were detected by immunofluorescence (IF), and the above matrix were stained by anti-Collagen II (ARG20787, Arigobio, China), anti-Collagen X (ARG59478, Arigobio), and anti-RGAG4 (HPA003652, Sigma-Aldrich). In addition, the above cartilage matrix was quantitatively analyzed by ImageJ software (National Institutes of Health, USA).

### 2.5. Detection of Mineralized Matrix Secreted by Chondrocytes

As shown in Section 2.4, chondrocytes were cultured in groups for 14 days; alkaline phosphatase (ALP) stain kit (A14353, Thermo Fisher scientific, USA) was used to stain and detected with IF. In the quantitative detection of ALP activity, 200 *μ*L Triton X-100 (X-100, Sigma-Aldrich, USA) was added to the cultured cells, and the lysed cell solution was detected by ALP Kit (ab83369, Abcam, USA). The detection process was carried out in strict accordance with the detection method of ALP kit. ALP activity was detected at the wavelength of 520 nm, and PBS solution was used as the blank control.

### 2.6. Articular Chondrocytes Activity Detection In Vitro

As shown in Section 2.4, chondrocytes were cultured in groups, and the cell activity detection in three groups would be performed by IF. After being cultured for 24 h, the cells were cleaned with PBS for 3 times and then fixed with 3% glutaraldehyde for 30 min. Alexa Fluor®488 Anti-Ki67 antibody [SP6] (ab281847, Abcam, USA) was used to label the active cells, and cell ability was observed by confocal microscope. Fluorescence spectrophotometer (WHF93, China) was used for fluorescence intensity test.

### 2.7. Articular Chondrocytes Apoptosis Evaluation In Vitro

As shown in Section 2.4, chondrocytes were cultured in groups for 24 h. After 3 times of cleaning with PBS, we added membrane breaker 0.3% Triton™ X-100 (X100, Sigma, USA) in the system and fixed it under 25°C for 15 min. Anti-caspase-3 antibody (ab32351, Abcam, USA) and annexin V (A7810, Sigma, USA) were added to mark apoptotic chondrocytes, and the reaction system were incubated avoiding light for 25 minutes. Flow cytometry (FCM) (Attune NxT, Thermo Fisher, USA) was performed to test the apoptotic chondrocytes.

### 2.8. Detection of Chondrocytes Migration

In order to detect the migration of chondrocytes cultured in groups as in Section 2.4, scratch test was used. After a scratch was made on the cell layer with a pipette gun, the chondrocytes at the scratch were washed out with PBS. After being cultured complete culture medium of human articular chondrocytes for another 24 h, the migration of chondrocytes was observed with a microscope, and the total number of migrating chondrocytes was calculated.

### 2.9. Statistical Methods

SPSS 22.0 and MedCalc software were adopted for statistical analysis. The quantitative data were described by *n* (%). The quantitative data was described by *x* ± *s*. A *t*-test was employed for intergroup comparison. *P* < 0.05 stands for striking difference.

## 3. Results

### 3.1. Chondrocytes Attraction Characteristics Detection of Gel

In the repair of osteoarthritis, attracting and migrating the cells in the surrounding tissue to the cartilage wound is of great significance to promote the repair of articular cartilage. If Gel can promote chondrocyte migration to the interior, it helps articular cartilage to be repaired from inside to outside. After 14 days of culture, the results showed that when the chondrocytes were inoculated on the Gel surface, fluorescence intensity of chondrocyte in each layer was different in layer by layer scanning (Figure 2(a)). The fluorescence intensity of FITC coupled with chondrocytes was the highest at the depth of 300-500 *μ*m (Figure 2(b)), indicating that Gel could help to attract chondrocytes to migrate to the interior and could be used as a cell matrix for chondrocytes regeneration.

### 3.2. Detection of Cartilage Matrix Secreted by Chondrocytes

In the repair of articular cartilage, collagen and GAGs present in the chondrocytes ECM are of great significance to improve the compressive and tensile properties of chondrocytes and promote chondrocytes proliferation. The results showed that compared with the control group and Gel group, Gel-nHA could stimulate chondrocytes to secrete more collagen type II (Figures 3(a)–3(d)). In terms of collagen type X generation, Gel-nHA could also stimulate chondrocytes to secrete more than control and Gel group (Figures 3(e)–3(h)). At the same time, chondrocytes secreted and produced more GAGs under the stimulation of Gel-nHA (Figures 3(i)–3(l)). The above results indicate that Gel-nHA can promote the secretion of collagen and GAGs, which was helpful to repair the cartilage.

### 3.3. ALP Activity Detection of Chondrocytes in Three Groups

The ability of Gel-nHA to induce chondrocyte mineralization is of great significance for repairing bone and cartilage interface and improving the connection between bone and cartilage. ALP staining showed that after 14 days of culture, the fluorescence intensity of chondrocytes cultured in Gel-nHA was higher than that in control and Gel group (Figures 4(a)–4(c)). Quantitative analysis showed that the ALP activity in Gel-nHA was 1.4 times higher than that in control group (Figure 4(d)). The above results suggest that Gel-nHA can further induce cartilage mineralization and provide a good foundation for the repair of bone cartilage interface.

### 3.4. Chondrocytes Activity and Apoptosis Evaluation in Three Groups

The activity of articular chondrocytes is very important for damaged articular cartilage repair, and anti-Ki-67 was used to detect cell activity. As shown in Figures 5(a)–5(d), the fluorescence intensity of Alexa Fluor®488 coupled with living chondrocytes cultured in Gel and Gel-nHA was significantly higher than that in pure medium, especially in Gel-nHA matrix, suggesting that Gel-nHA has good compatibility with chondrocytes, and the addition of nHA can further improve the proliferation activity of chondrocytes. The apoptosis degree of articular chondrocytes can indirectly reflect its cartilage repair ability. In this study, apoptotic articular chondrocytes were labeled with anti-caspase-3 and annexin V. FCM showed that compared with control group (Figure 5(e)), less apoptosis cells were found in Gel and Gel-nHA group, especially in Gel-nHA group (Figures 5(f) and 5(g)), and the quantitative evaluation also showed the same results (Figure 5(h)). The above results mean that Gel can provide a good matrix for chondrocyte survival, and nHA can further reduce the apoptosis of chondrocytes.

### 3.5. Chondrocytes Migration Evaluation in Three Groups

In the repair of articular cartilage, the migration activity of chondrocytes can significantly improve its repair effect. In Gel and Gel-nHA matrix, the migration activity of chondrocytes was significantly higher than that of the control group, especially in Gel-nHA matrix (Figure 6), suggesting that Gel can provide a good cell substrate for chondrocyte migration in vitro and nHA can further promote the migration of chondrocytes.

## 4. Discussion

With the aging of population, the incidence rate of osteoarthritis has been increasing year by year, and the main symptom is degenerative injury of articular cartilage [18]. As one of the most frequently used joints in human body, long-term weight-bearing can easily lead to talus cartilage wear in ankle joint, resulting in ankle swelling, pain, and restricted activity disorder, which will seriously affect the life quality of patients [19]. However, the poor blood supply in cartilage tissue hinders the self-repair of articular cartilage. At this stage of treatment, symptomatic pain relief treatment and improvement of joint activity function are mainly carried out, but the produced articular cartilage is mainly composed of type I collagen fibers [20], which have relatively poor compressibility and elasticity. With the development of biotechnology, more and more new materials have been used in the treatment of articular cartilage injury, such as Gel, which has good histocompatibility and natural ECM like structure [21]. Therefore, if injected into the joints, Gel can encapsulate the irregular cartilage degradation areas, so as to support the migration and proliferation of chondrocytes [22]. It is expected to become a new method for the treatment of osteoarthritis.

Gel has low viscosity and good fluidity, so that they can enter the articular cavity through injection and fully integrate with the defective cartilage [23]. Secondly, the ECM like structure can encapsulate chondrocytes and collagen in the mesh, which is conducive to cell proliferation. Furthermore, due to the strong water retention ability, Gel can better maintain the proliferation activity of chondrocytes than other scaffold [24, 25]. Its good biocompatibility and degradability can make it well compatible with surrounding tissues and effectively reduce the occurrence of inflammatory reaction [26, 27]. Therefore, Gel is a good tool for transporting biomaterials. nHA, as the main inorganic salt in bone, can effectively promote bone growth and repair and prevent osteoporosis [28]. In recent years, some studies have found that nHA can also induce the differentiation of chondrocytes and promote the secretion of chondrocytes ECM, such as collagen and GAGs [29, 30]. Therefore, studying the repair effect of Gel-nHA composite scaffold in joint cartilage injury is of great significance for improving the curative effect of osteoarthritis.

In the treatment of osteoarthritis, it is important to promote the migration of chondrocytes from surrounding tissues to damaged cartilage. In the study of physicochemical properties of Gel, we found that the chondrocytes distributed in different depths, and the fluorescence intensity was the highest at the depth of 300–500 *μ*m in Gel, suggesting that Gel has the potential of inducing and attracting chondrocytes. This is mainly related to the good affinity between Gel and chondrocytes, which can provide a good environment for the proliferation of chondrocytes. In addition, Gel's natural ECM-like structure is conducive to the adhesion of chondrocytes and guides them to migrate to the skeleton to secrete matrix and better maintain their phenotype of chondrocytes, which helps it as an acellular matrix scaffold for chondrocyte regeneration.

ECM helps to maintain cell viability and effectively promote cell differentiation, adhesion, and migration. During the process of cartilage repair, promote secretion of collagen and GAGs and deposit in Gel to form cartilage ECM, which is of great significance. It was found that the addition of nHA could effectively promote the secretion of collagen type II and GAGs, which would help to promote the formation of cartilage and increase the compressibility and extensibility of new cartilage. In addition, maintaining the integrity of bone cartilage interface is also an important part of joint repair. Bone cartilage interface is mainly formed by calcified cartilage, which is of great significance in inhibiting the invasion of bone to cartilage. It was found that nHA helped to improve the mineralization ability of articular chondrocytes and stimulate the secretion of collagen type X, which could further promote the formation of calcified cartilage, so as to maintain the integrity of bone cartilage interface. Guo et al. [9] et al. found that in the rabbit model of knee cartilage defect, the use of polyvinyl alcohol/nanohydroxyapatite/polyamide 66 could effectively promote the generation of type II collagen, thus better promoting the repair of articular cartilage. It is consistent with the results of this study.

The proliferation activity of chondrocytes is closely related to cartilage repair. It was found that in the Gel, the proliferation viability of chondrocytes was significantly improved. In addition, the addition of nHA could further decrease the apoptosis of chondrocytes. This was mainly related to Gel biological scaffold which promoted cell adhesion, differentiation, and migration. In addition, nHA could stimulate the secretion of collagen and GAGs, so as to better promote the repair of talus cartilage. However, this study mainly stays in the experimental stage, and there is no animal osteoarthritis model to further evaluate the comprehensive performance of Gel-nHA, which needs to be further improved in later research, so that it can be used in the repair of articular cartilage injury in clinic as soon as possible.

## 5. Conclusion

In this study, we designed a new biopolymer scaffold for the repair of talus cartilage, mainly composed of Gel and nHA. We found that the Gel could guide the migration of chondrocytes, and could be used as an acellular matrix scaffold for chondrocyte regeneration. After adding nHA, it helped to stimulate chondrocytes to secrete cartilage matrix, such as collagen and GAGs, so as to better maintain the proliferative activity of chondrocytes and increase the elasticity and stretch of new cartilage. At the same time, nHA could induce the mineralization of chondrocytes, and the secretion of collagen type X could further induce the formation of calcified cartilage, so as to maintain the integrity of bone cartilage interface and better repair the damaged talus articular surface. Therefore, the Gel-nHA scaffold is expected to become an effective method for talus cartilage repair in the future.

## Figures and Tables

**Figure 1:** Schematic of the assembly process for Gel-nHA and its mechanism.

**Figure 2:** Internal migration of chondrocytes into Gels: (a) distribution of chondrocytes under confocal microscope (the depth of each layer is 50 *μ*m), ×40; (b) quantitative distribution of total fluorescence intensity of FITC coupled with chondrocytes.

**Figure 3:** Detection of cartilage matrix secreted by chondrocytes. (a–c) Anticollagen II expression in control, Gel, and Gel-nHA group, ×20. (d) Quantitative analysis of collagen type II. (e–g) Anticollagen X expression in control, Gel, and Gel-nHA group, ×20. (h) Quantitative analysis of collagen type X. (i–k) Anti-RGAG4 expression in control, Gel, and Gel-nHA group, ×20. (l) Quantitative analysis of GAGs. ∗*P* < 0.05.

**Figure 4:** Detection of mineralization ability of chondrocytes. (a–c) ALP fluorescent staining in control, Gel, and Gel-nHA group, ×20. (d) Quantitative evaluation of ALP relative activity in control, Gel, and Gel-nHA group. #*P* > 0.05, ∗∗*P* < 0.01.

**Figure 5:** Chondrocytes activity and apoptosis assessment. (a) Anti-Ki67 expression pattern in control group, ×20. (b) Anti-Ki67 expression pattern in Gel group, ×20. (c) Anti-Ki67 expression pattern in Gel-nHA group, ×20. (d) Fluorescence intensity quantitative evaluation of Alexa Fluor®488 coupled with living chondrocytes in control, Gel, and Gel-nHA group. (e) FCM result of chondrocytes in control group. (f) FCM result of chondrocytes in Gel group. (g) FCM result of chondrocytes in Gel-nHA group. Quantitative evaluation of apoptotic chondrocytes in control, Gel, and Gel-nHA group. ∗*P* < 0.05.

**Figure 6:** Chondrocytes scratch test. (a) Chondrocytes in control group, ×10; (b) chondrocytes in Gel group, ×10; (c) chondrocytes in Gel-nHA group ×10; (d) quantitative evaluation of migration cells in control, Gel, and Gel-nHA group. ∗∗*P* < 0.01 and ∗*P* < 0.05.

## Data Availability

The labeled datasets used to support the findings of this study are available from the corresponding author upon request.
